This article has been retracted.

# Analysis of PICC Based on Dysfunction Module Personalized Nursing Treatment in Chemotherapy of Advanced Esophageal Cancer

**DOI:** 10.1155/2021/8997915

**Published:** 2021-07-21

**Authors:** Qixin Zhang, Aili Qian, Weifen Chen

**Affiliations:** ^1^Department of Anorectal Surgery, Jinan People's Hospital, Laiwu 271100, Shandong, China; ^2^Hospital Infection Management Office of Jinan No. 4 People's Hospital, Jinan 250000, Shandong, China; ^3^The Affiliated Hospital of Qingdao University, Qingdao 266000, Shandong, China

## Abstract

Esophageal cancer is a common malignant tumor in some countries and regions in the world, which threatens the health of people all over the world. Due to esophageal cancer, about 400,000 people die every year. Among them, the number of cases and deaths of esophageal cancer in our country accounts for about 50% of the world. This article aims to study the clinical efficacy of PICC catheterization in the chemotherapy of advanced esophageal cancer based on the dysfunction module. For patients with advanced esophageal cancer, traditional surgery is still difficult to achieve satisfactory results. Therefore, in order to improve the therapeutic effect of esophageal cancer and obtain a higher clinical effective rate and pathological complete remission rate, it is necessary to explore a new comprehensive treatment model. In this paper, the theoretical knowledge of PICC is described in detail from the concept, advantages, and indications of PICC, and the SPSS statistical method is proposed. The SPSS statistical model, mean test, two-independent sample *t*-test, and regression analysis jointly explain the application principles and methods of SPSS statistical methods. After selecting the experimental subjects, the 180 eligible patients with esophageal squamous cell carcinoma were divided into two groups, each with 30 patients with stage II esophageal cancer, 30 patients with stage III esophageal cancer, and 30 patients with stage IV esophageal cancer. Grouping according to different variables, real-time recording of data, and SPSS statistical method to analyze the experimental data, the experimental results of this article show that the nursing satisfaction of the observation group is 92.2%, which is significantly higher than the 56.7% of the control group, so it can be seen that PICC plays an important role in the personalized care and treatment of advanced esophageal cancer.

## 1. Introduction

In recent years, with the continuous rapid development of economy and technology, the pace of human life is accelerating, and the incidence of cancer and other diseases is also increasing. Cancer is a chronic disease, which is affected by many factors such as age and gender. It is in this situation that cancer treatment and nursing intervention have become an important part of clinical research. In addition to basic hospital care, targeted nursing interventions should also be carried out according to the type of cancer that cancer patients have. Esophageal cancer is one of the most common gastrointestinal cancers in China, and Hebei Province in northern China has one of the highest incidences of esophageal cancer. Compared with the past, the latest developments and advances in medical technology have improved the survival rate of patients, but the prognostic effect of esophageal cancer is still very poor. Traditional nursing methods can no longer meet the needs of patients, especially in the process of PICC for patients. In PICC, care must be taken to avoid shedding and other complications, and related issues such as the puncture rate should be reduced. The care of PICC in cancer patients has also attracted the attention of many researchers.

Due to the high degree of local and distant recurrence and metastasis of esophageal cancer after surgical resection, most patients are in the middle and late stage at the first visit. Therefore, in addition to actively improving the effect of early diagnosis and treatment of esophageal cancer, more attention needs to be paid to improving the treatment rate of patients with advanced esophageal cancer. At present, chemotherapy is the main treatment for most diseases. Most chemotherapeutic drugs require intravenous injection, but repeated venipuncture will destroy superficial veins, increase patient suffering, and greatly increase the burden on nursing staff. Peripheral vein implantation of PICC is a common method of intravenous injection, which can prevent the irritation of chemotherapeutic agents to venous blood vessels. During chemotherapy, high concentrations of chemotherapeutics will increase vascular permeability and drug overflow, which will affect surrounding tissues and easily cause new diseases. PICC is very useful for the treatment of patients, which can avoid iatrogenic Shanghai.

Since the rapid spread of the Internet of Things (IoT) as a new communication paradigm, KimB has conducted research on various applications. In particular, interest in smart medical systems is rising. In an intelligent medical system, many medical devices are distributed in popular areas such as stations and medical centers, and such high-density medical device distribution can cause severe communication performance degradation, which is called a coexistence problem. However, when a coexistence problem occurs in the smart medical system, the reliable transmission of the patient's biological information may not be guaranteed, and the patient's life may be endangered [1]. In the developing world, reliable data on economic livelihoods are still scarce, which hinders efforts to study these results and formulate policies to improve them. Here, Jean demonstrates an accurate, cheap, and scalable method for estimating personal consumption and wealth based on high-resolution satellite images. It demonstrates how to use research and satellite data from five African countries to train a cohesive neural network to recognize image features, and these image features can explain up to 75% of local level economic changes. It also shows how to apply powerful machine learning techniques with limited training data, showing that there are wide-ranging potential applications in many scientific fields. However, due to the unbalanced economic level, the actual effect is not very satisfactory [2]. The discovery of new materials can bring about tremendous social and technological progress. In this case, it is computationally tricky to fully explore the huge space of potential materials. Here, Benjamin reviews the method of realizing reverse design, which aims to discover tailor-made materials from the starting point of specific required functions. The latest developments in the rapidly developing field of artificial intelligence (mainly a subfield of machine learning) have led to the exchange of ideas, in which methods for reverse molecular design have been proposed and quickly adopted. Among them, the deep-level generation model has been applied to a variety of material categories: rational design of expected drugs, ways to synthesize organic compounds, optimization of photovoltaic cells and redox flow batteries, and various other solid materials. However, the stability of the material is not very good, leading to errors in the results [3, 4].

The innovations of this article include the following: (1) the use of scientific statistical methods to improve the validity and credibility of the final experimental results; (2) in order to improve the clinical efficacy of patients with esophageal cancer during chemotherapy, the PICC-based personality detailed analysis and research on the clinical application of chemical nursing in patients with esophageal cancer.

## 2. Individualized Nursing Treatment Methods in Chemotherapy of Advanced Esophageal Cancer

### 2.1. Introduction to PICC

#### 2.1.1. The Basic Concept of PICC

The full name of PICC is Peripherally Inserted Central Venous Catheter [5, 6]. PICC is a combination of the first letters of its full English name. The PICC tube is a catheter that is punctured and intubated from the peripheral vein on the arm and then passes through the axillary vein, subclavian vein, and innominate vein in the direction of the blood vessel and finally inserts the tip of the catheter into the superior vena cava [7, 8]. The schematic diagram of the PICC catheter in the body is shown in Figure 1.

#### 2.1.2. Advantages of PICC

1. It reduces the pain caused by repeated puncture.
2. It protects blood vessels and avoid complications caused by drug extravasation.
3. Continuous long-term venous access can ensure the smooth progress of various treatments and rescues.
4. It reduces patients' vomiting and white blood cell depletion degree of the drug is also reduced, and the drug is used to reduce the venous residence time, and it is directly metabolized and excreted through the blood to reduce irritation.
5. In the jugular vein, venous vein perforation, and femoral vein perforation, PICC is easy. Use it and succeed with the help of B. The nurse can complete this operation independently. The operation method is simple and easy to use. It is not restricted by time and place, and the work efficiency is also improved.
6. The material is very soft, blends perfectly with the limbs, and is not easy to break. The catheter itself is anti-inflammatory. There are anticoagulant and antithrombotic effects, especially the front opening of PICC with 3D valve. When the valve is not injected and closed, it can effectively prevent blood backflow and cause tube blockage or air blockage, greatly reducing complications after catheter placement and extending the catheter retention time by 1-2 years.
7. After the catheter is inserted, it will not affect the daily life of the patient, such as eating, dressing, washing face, brushing teeth, and bathing.
8. PICC puncture will only show mild trauma, long retention time, and low infection rate. Long-term use can meet the various needs of cancer patients undergoing chemotherapy [9–11].

#### 2.1.3. PICC Indications and Applications

1. It is suitable for patients with long-term intravenous infusion.
2. It is suitable for patients who cannot easily enter peripheral veins.
3. It is suitable for patients who inject irritating and corrosive drugs.
4. It is suitable for injection of parenteral nutrition solutions or hypertonic or viscous patients with liquids (such as mannitol).
5. It is suitable for patients who need repeated blood transfusion or repeated blood drawing.
6. It can be home nutrition or treatment, suitable for patients who have received treatment [12].

### 2.2. PICC-Based Personalized Nursing Treatment in Chemotherapy of Advanced Esophageal Cancer

With the aging of our country, the number of elderly patients with esophageal cancer will gradually increase in the near future. Esophagectomy is the treatment of choice for patients with locally advanced esophageal cancer. But for many elderly patients, because they not only have organ failure, but also have a variety of underlying diseases and other factors, many elderly people are unwilling to undergo surgery. Therefore, radiotherapy and chemotherapy have become the first choice for the treatment of esophageal cancer in the elderly [13].

Many problems are prone to occur during PICC catheter treatment. For example, if the catheter is blocked, it will stay in the patient's body for a short time, which will affect the healing effect. Therefore, individualized care is required during the treatment of PICC catheter patients [14, 15].

Before inserting the catheter, the nursing staff must accurately understand the patient's illness information and record the patient's daily condition before taking care of the patient. Before performing the catheterization, the nursing staff should explain the PICC catheterization methods, precautions, adjustment points, and complications that may occur during the catheterization of the patient and his family in easy-to-understand terms [16]. Let the patient and his family fully understand the purpose and risks of PICC intubation, and after understanding the treatment of PICC intubation, ask the patient or family member to sign a consent form. Before intubation, the patient can be put into a state of complete anesthesia to reduce the patient's tension. Thoroughly evaluate the various physiological parameters of the patient to reduce the pain during catheterization, and select the appropriate vein for catheterization [17, 18].

After inserting the catheter, first determine the patient's venipuncture position, and then assess the patient's risk of venipuncture success rate. After evaluation, if the success rate of puncture is not high, you need to reselect a suitable puncture site. After the puncture risk assessment, the patient's arm to be operated on was abducted by 90°, the patient was asked to lie down, and the distance from the patient's puncture point to the right sternal clavicular joint was measured. Measure the circumference of the arm 10 cm above the cube light, and expose the puncture site to the patient for regular disinfection [19]. Inform the patient not to move during the puncture to avoid misalignment of the puncture. After the puncture is completed, it should be sterilized again and a compression bandage should be used to prevent bleeding at the puncture site. During this period, the nursing staff should keep the nursing records during the PICC operation, such as position, length and arm circumference, catheter insertion time, and catheter perforation bleeding [20].

After placing the catheter, pay special attention to whether the position of the catheter tip has changed after the PICC is placed. When puncturing the patient's puncture site, choose a well-ventilated dressing and change it regularly. When changing the bandage, make sure that the catheter at the puncture site is red and swollen and not misplaced. Observe the blood at the puncture site before and after the incision, and disinfect the puncture site to prevent infection. When removing the catheter, please hold down for 3 minutes to avoid bleeding after moving the catheter. Then, within three days of inserting the tube, the patient was instructed not to do obvious exercises and to take several hemostatic drugs when needed. Strictly comply with aseptic technique requirements during patient intubation. Before injecting the patient, push the catheter with saline to prevent the catheter from being blocked. After the injection, an intravenous injection is also performed to flush the drug into the catheter to prevent the catheter from being blocked [18, 21].

### 2.3. SPSS Statistical Methods

#### 2.3.1. SPSS Statistical Model

In the personalized care and treatment methods in the chemotherapy of advanced esophageal cancer, the logarithmic model, exponential smoothing model, and RIMA product model are used to predict the experimental data of esophageal cancer patients in the observation group and the control group [22, 23]. The specific methods are as follows:

1. Logarithmic model:
2. The logarithmic model is a curvilinear regression prediction model in SPSS software. It is one of the most commonly used time series forecasting methods. It is mainly used in the process of irregularly changing time series forecasting, but the available time series are relatively short.
3. Exponential smoothing model:
4. In the process of model construction, there are four basic parameters: traditional configuration, voltage parameters, period parameters, and voltage correction parameters, which correspond to *α*, *γ*, *δ*, and *π*, respectively. In addition to the correction parameters, the other three parameters can also be integrated into the weights of the most recently observed data. The price ranges from 0 to 1. The closer the value is to 1, the higher the weight of the observation is. The data mainly controlled by *π* shows a downward trend, with weights ranging from 0 to 1, but never equal to 1. The closer the value is to 1, the faster the voltage drop rate changes.
5. ARIMA model:
6. The model mainly uses regressors and moving averages to achieve prediction goals. It is mainly used for data processing that changes greatly over time. Therefore, it consists of many submodels called self-development AR, the sum is I, and the moving average is MA. AR and MA are set to *p* and *q*, respectively, and the frequency of data difference is set to *d*. It can be converted to the following formula:

(1) $$\begin{array}{c} \phi \left(W\right)\nabla^{d}x_{1}=\theta \left(W\right)e_{1}. \end{array}$$

Here, *W*, ∇^*d*^, *ϕ*(*W*), and *θ*(*W*), respectively, correspond to the postshift operator, postdifference operator, autoregressive operator, and moving average operator. The more orders in the equation, the more types and numbers of parameters involved in the ARIMA model.

SPSS is widely used in teaching evaluation. In addition to statistical analysis of various types of problems, reliability metrics can also be used to determine whether the test can reflect the actual level and analyze various related factors that can be quantified. Combined with SPSS analysis, a more scientific and rigorous conclusion can be drawn.

#### 2.3.2. Mean Test

The mean test is more practical when calculating the comprehensive descriptive statistics of the specified variables. In the analysis process, descriptive statistics need to be calculated, so the average test is used [24]. When outputting, output: a series of univariate descriptive statistics such as mean, standard deviation, variance, and skewness:

(1) Average: arithmetic average; the sum is divided by the number. The calculation formula of the average value is
  (2) $$\begin{array}{c} \bar{Y}=\frac{\sum_{i=1}^{n}Y_{i}}{n}. \end{array}$$
(2) Standard deviation: Karl Pearson uses statistical standard deviation, which is usually used to measure the degree of statistical distribution, that is, the degree of dispersion between individuals in the group. In this study, there is a great reference for analyzing sample data. The calculation formula of standard deviation is
  (3) $$\begin{array}{c} s=\sqrt{\frac{\sum_{i=1}^{n}{\left(Y_{i}-\bar{Y}\right)}^{2}}{n-1}}. \end{array}$$
(3) Variance: the square of the standard deviation, like the standard deviation, describes the distance of the variable from its expected value. The calculation formula of variance is
  (4) $$\begin{array}{c} s^{2}=\frac{\sum_{i=1}^{n}{\left(Y_{i}-\bar{Y}\right)}^{2}}{n-1}. \end{array}$$

#### 2.3.3. Two Independent Samples' *t*-Test

The *t-*test of two independent samples is a statistical technique used to determine whether there is a significant difference between two independent samples [25]. Only statistical testing can determine whether the difference between the two average scores is significant and analyze the data objectively.

Its main steps are as follows.

Step 1: perform a significant difference test on the means of the two populations. Assuming that the mean values of the two samples are equal, *I*_0_ is *μ*_1_ = *μ*_2_; assuming that the mean values of the two samples are not equal, *μ* 1 ≠ *μ* 2.
Step 2: if the null hypothesis holds, the independent sample *t-*test will use the statistic *t*. Specifically, it can be divided into two situations. If the sample differences are equal, the *t* statistic is defined as
  (5) $$\begin{array}{c} t=\frac{\left(\bar{Y_{1}}-\bar{Y_{2}}\right)-\left(\mu_{1}-\mu_{2}\right)}{S_{\omega }\sqrt{\left(1/n_{1}+1/n_{2}\right)}}. \end{array}$$
Among them,
  (6) $$\begin{array}{c} S_{\omega }^{2}=\frac{\left(n_{1}-1\right)S_{1}^{2}+\left(n_{2}-1\right)S_{2}^{2}}{\left(n_{1}+n_{2}\right)-2}, \end{array}$$
where *n*_1_ and *n*_2_ are the two sample sizes and *s*_1_ and *s*_2_ are the standard deviations of the two samples. This statistic obeys the *t* distribution with (*n*_1_+*n*_2_) − 2 degrees of freedom. When the sample variances are not equal, the *t* statistic is defined as
  (7) $$\begin{array}{c} t=\frac{\left(\bar{Y_{1}}-\bar{Y_{2}}\right)-\left(\mu_{1}-\mu_{2}\right)}{\sqrt{\left(S_{1}^{2}/n_{1}+S_{2}^{2}/n_{2}\right)}}. \end{array}$$
When analyzing the output data of the *t*-test of two independent samples, first, you need to run a variance consistency test, and then you can check whether the two population means are the same.
Step 3: if the given null hypothesis is true, the observation value of statistical test and its *p* value can be obtained by replacing the *μ*_1_ − *μ*_2_ part of the *t* statistic with 0.
Step 4: make statistical conclusions based on the significance level. If the *p* value is less than 0.05, there is a significant difference between the two population means. On the contrary, there is no significant difference [26–28].

#### 2.3.4. Regression Analysis

In statistics, regression analysis is a statistical analysis method used to determine the quantitative relationship between two or more variables. Regression analysis can be divided into simple regression analysis and multiple regression analysis, depending on the number of variables involved. According to the number of dependent variables, it can be divided into single regression analysis and multiple regression analysis. According to the independent variables between types, dependent variables can be divided into linear regression analysis and nonlinear regression analysis.

(1) Multiple linear regression:
The independent variable corresponds to the *X* axis in the graph, and the dependent variable is the response variable, which corresponds to the *Y* axis. Multiple linear regression has many independent variables and is linearly related to the dependent variable. The mathematical model of multiple linear regression is
  (8) $$\begin{array}{c} y=\left(\beta_{0}+\beta_{1}x_{1}+\beta_{2}x_{2}+\beta_{k}x_{k}\right)+\varepsilon , \end{array}$$
where *β*_0_, *β*_1_, *β*_2_,…, *β*_*k*_ is *k* + 1 unknown parameters, *β*_0_ is regression constant, and *β*_0_, *β*_1_, *β*_2_,…, *β*_*k*_ is called regression coefficient; *y* is called the explained variable; *x*_1_, *x*_2_,…*x*_*k*_ is *k* explanatory variables; and *ε* is random error. The calculation of regression coefficients is extremely complicated, but as long as the observations are input in SPSS, all parameters can be obtained. After integration, multiple linear empirical equations can be obtained:
  (9) $$\begin{array}{c} \overset{\wedge }{y}=\overset{\wedge }{\beta_{0}}+\overset{\wedge }{\beta_{1}}x_{1}+\overset{\wedge }{\beta_{2}}x_{2}+\cdots +\overset{\wedge }{\beta_{k}}x_{k}. \end{array}$$
(2) Test of regression equation:
  ① Test of correlation coefficient:
  After obtaining the linear regression equation, it is necessary to analyze the fitting effect of the linear regression equation. The correlation coefficient is often used to indicate the degree of agreement between the equation to be sought and the actual equation:
    (10) $$\begin{array}{c} R^{2}=\frac{\text{SSR}}{\text{SST}}=1-\frac{\text{SSE}}{\text{SST}}=1-\frac{\sum \left({\left(y-\overset{\wedge }{y}\right)}^{2}\right)}{\sum {\left(y-\bar{y}\right)}^{2}}. \end{array}$$
    Here, *SSR* is the regression sum of squares, SSE is the residual sum of squares, and *SST* is the total deviation of squares. The range of *R*^2^ is 0∼1; the closer to 1, the better the fit. As the number of independent variables increases, *R*^2^ will increase and must be adjusted. The adjusted *R*^2^ is
    (11) $$\begin{array}{c} {\bar{R}}^{2}=1-\frac{\text{SSE}/\left(n-k-1\right)}{\text{SST}/\left(n-1\right)},\\ =1-\frac{\text{SSE}}{\text{SST}}•\frac{n-1}{n-k-1},\\ =1-\left(1-R^{2}\right)\frac{n-1}{n-k-1}. \end{array}$$
  ② *F* test:
  The statistic *F* can also reflect the degree of fit of the adjusted regression equation. Combining equation *R*^2^ to transform statistical equation *F*, formula (12) is obtained. From the equation, we can see that when the good fit of the regression equation is very high, the *F* statistic is the most obvious.
    (12) $$\begin{array}{c} F=\frac{R^{2}/k}{\left(1-R^{2}\right)/\left(n-k-1\right)}. \end{array}$$

#### 2.3.5. Correlation Analysis

Correlation analysis is a statistical analysis method used to investigate the correlation of two or more random variables at the same location. For example, the relationship between human height and weight and the relationship between relative humidity and rainfall are all aspects that can be analyzed and researched.

(1) Correlation coefficient:
The main purpose of correlation analysis is to study the closeness of the relationship between variables. Correlation can be divided into positive correlation, negative correlation, and irrelevance. Depending on the characteristics of the data, different correlation coefficients are usually used, denoted by *r*. The following are three commonly used correlation coefficients:
  ① Pearson correlation coefficient:
  The Pearson correlation coefficient is also the linear correlation coefficient, and its calculation formula is
    (13) $$\begin{array}{c} r=\frac{\sum_{i=1}^{n}\left(Y_{i}-\bar{Y}\right)\left(X_{i}-\bar{X}\right)}{\sqrt{\sum_{i=1}^{n}{\left(Y_{i}-\bar{Y}\right)}^{2}}\sqrt{\sum_{i=1}^{n}{\left(X_{i}-\bar{X}\right)}^{2}}}. \end{array}$$
  Among them, *n* is the sample size, and *x*_*i*_ and *y*_*i*_ are the corresponding sample values of the two variables. Its *t*-test statistic is
    (14) $$\begin{array}{c} t=\frac{\sqrt{n-2}}{\sqrt{1-r^{2}}}. \end{array}$$
  Among them, the *t* statistic obeys the *t* distribution with *n* -2 degrees of freedom.
  ② Spearman rank correlation coefficient:
  The Spearman rank correlation coefficient does not require the distribution of initial variables and has a wide range of uses. The calculation formula of Spearman rank correlation coefficient is as follows:
    (15) $$\begin{array}{c} r_{s}=\frac{\sum_{i=1}^{n}\left(R_{i}-\bar{R}\right)\left(S_{i}-\bar{S}\right)}{\sqrt{\sum_{i=1}^{n}{\left(R_{i}-\bar{R}\right)}^{2}\sum_{i=1}^{n}{\left(S_{i}-\bar{S}\right)}^{2}}}=1-\frac{6\sum_{i=1}^{n}d_{i}^{2}}{n\left(n^{2}-1\right)}. \end{array}$$
  Among them,
    (16) $$\begin{array}{c} \bar{R}=\frac{1}{n}\sum_{i=1}^{n}R_{i},\bar{S}=\frac{1}{n}\sum_{i=1}^{n}S_{i}. \end{array}$$
  The *L* statistic of Spearman's rank correlation coefficient is
    (17) $$\begin{array}{c} L=r\sqrt{n-1}. \end{array}$$
  ③ Kendall rank correlation coefficient:
  Kendall's rank coefficient is a measure of two variables or degree of relationship among variables. The calculation formula of Kendall's rank correlation coefficient is
    (18) $$\begin{array}{c} r=\frac{2\left(V-W\right)}{n\left(n-1\right)}. \end{array}$$

The *D* statistic of Kendall rank correlation coefficient is

(19) $$\begin{array}{c} D=\tau \sqrt{\frac{9n\left(n-1\right)}{2\left(2n+5\right)}.} \end{array}$$

The correlation coefficient *r* represents the linear relationship between two variables. If *r* is greater than 0, the two variables have a positive correlation; if *r* is less than 0, both variables have a negative correlation: 1 and −1. The closer the absolute value of *r* is to 1, the greater the degree of linear relationship between the two variables. The correlation coefficient *r* and its degree of correlation are shown in Figure 2:

  Positive correlation: this means that the two variables change in the same direction, and the slope of the data tangent to the curve is always greater than zero.
  Negative correlation: it is the opposite of positive correlation and refers to two variables in opposite directions, and the tangent slope of the data curve is always less than zero; that is, the correlation coefficient is less than zero.

## 3. PICC's Personalized Nursing Treatment Experiment in the Chemotherapy of Advanced Esophageal Cancer

### 3.1. Experimental Goals of Personalized Nursing Treatment in Chemotherapy for Advanced Esophageal Cancer

The radiotherapy oncology group (RTOG) trial has passed randomized and nonrandomized phase III trials, and the comparison shows that, in the 5-year survival rate, radiotherapy and chemotherapy are significantly better than radiotherapy alone (the randomized group of radiotherapy and chemotherapy compared with radiotherapy alone is 26% vs. 0%, compared with radiotherapy alone in the nonrandomized group, 14% vs. 0% of radiotherapy and chemotherapy), which established that the combination of radiotherapy and chemotherapy has obvious advantages over radiotherapy alone in the choice of treatment for esophageal cancer. However, this radiotherapy and chemotherapy program has more advantages. There are large acute chemical toxic side effects, but no treatment has been devoted to elderly patients with esophageal cancer. At this stage, there is no specific study to determine the standard treatment strategy for elderly patients with esophageal cancer. In order to further clarify the role of radiotherapy and chemotherapy alone in elderly esophageal cancer, this study collected 180 patients with advanced esophageal cancer who are over 70 years old for a retrospective study to provide better support for clinical practice.

### 3.2. Selection of Experimental Subjects for Personalized Nursing Treatment in Chemotherapy of Advanced Esophageal Cancer

#### 3.2.1. Patient Enrollment Conditions

Patient enrollment conditions were the following: (1) age older than 70 years; (2) pathologically confirmed patients with esophageal cancer; (3) all patients being were treated for the first time (surgical resection could not be or refused); (4) ECOG score ≤ 2 points; no contraindications to radiotherapy and chemotherapy; (5) relevant radiotherapy and chemotherapy consent form; (6) no history of other malignant tumors; (7) complete case data.

#### 3.2.2. Patient Exclusion Conditions

Exclusion criteria were the following: (1) age less than 70 years; (2) pathologically confirmed patients with nonesophageal cancer; (3) having undergone surgery, radiotherapy, and chemotherapy; (4) having radiotherapy and chemotherapy contraindications; (5) having a history of other malignant tumors; (6) lacking complete case data; (7) chemotherapy greater than 4 cycles; (8) giving up treatment; (9) pregnant and lactating women; (10) having conventional, three-dimensional conformal radiotherapy; (11) early stage I esophageal cancer; (12) occurrence of distant metastasis.

#### 3.2.3. Clinical Characteristics of the Patients

180 patients with esophageal squamous cell carcinoma who met the enrollment conditions were divided into two groups: each group had 30 patients with stage II esophageal cancer, 30 patients with stage III esophageal cancer, and 30 patients with stage IV esophageal cancer, and the pathology of all patients in the group was of the same type. The balance between the two groups of patients is good, and the statistical analysis of the baseline data shows that the experiment is comparable.

#### 3.2.4. Clinical Staging

The clinical staging of all enrolled patients was based on the clinical staging standard for nonsurgical treatment of esophageal cancer. For some patients who cannot be covered by *N* stage and clinical stage, please refer to the analysis of the safety and efficacy of radiotherapy for advanced esophageal cancer of patients who are over 70 years old compared with radiotherapy alone. In addition, a comprehensive physical examination is required. We will confirm the staging results through abdominal B-ultrasound, whole-body ECT, CT scan, and PET-CT.

### 3.3. Grouping of Experimental Subjects for Personalized Nursing Treatment in Chemotherapy of Advanced Esophageal Cancer

The observation group can also be referred to as the experimental group to carry out PICC nursing work. In the process of nursing work, nursing staff should always observe the patient's physiological changes to reduce the patient's stress response. It should also be noted that the exposed length of the patient's catheter should be controlled. It should not be too short or too long. It is generally three to five centimeters. This is because the external catheter is too long, exposed, and easy to wrap, so it is difficult to fix. Every time you perform catheter maintenance, carefully observe whether there is bleeding, sweating, pain, and itching at the puncture site, whether there is any secretion around the puncture site, and whether the veins are rope-shaped. Choose a suitable skin disinfectant for puncture and maintenance. Do not use rubbing alcohol to clean the wound to prevent excessive irritation and difficulty in healing the wound. After the disinfectant is completely dry, use a sterile, breathable, good viscosity, and nonallergenic film. Nontensioned accessories are used, and the conduit and connector are placed in a semiarc shape. Rotation, folding, or angle formation is strictly prohibited. Attention should also be paid to effective publicity and education of patients, instructing patients to perform appropriate exercises, etc. to avoid strenuous upper limb activities and excessive abduction, lifting, rotation, and frequent bending and stretching activities during activities. The arm with a tube can be used for some active exercises, such as relaxing your fists.

The control group took routine infusion care.

## 4. Experimental Analysis of Personalized Nursing Treatment in Chemotherapy of Advanced Esophageal Cancer

### 4.1. Personalized Nursing Treatment Content

#### 4.1.1. On Diet

The cancer itself reduces the various normal functions of the patient and consumes the patient's diet. Therefore, attention should be paid to timely supplementation of various nutrients in the patient's daily diet to increase the patient's resistance. Eat foods with high protein, calories, and digestibility, and eat small and frequent meals to avoid gastrointestinal discomfort. Nursing staff need to create a good treatment environment for patients, and teach patients to relax, so that patients can respond to challenges with a positive attitude.

#### 4.1.2. Psychology

Cancer not only harms human health, but also exerts psychological pressure on cancer patients. Because some patients cannot fully understand cancer, they believe that all cancers are incurable. After cancer is discovered, it will exert pressure and cause many psychological problems, such as fear and anxiety. According to research on relevant data, patients' unhealthy feelings (such as neuroticism and stress) gradually reduce their confidence in disease treatment, which is a major stumbling block for patients in treatment and affects their physical recovery. At the same time, patients tend to feel that their condition is getting worse during the treatment process, which increases the patient's own psychological burden and affects the treatment effect. Therefore, it is very important to provide patients with extensive psychological care. Taking into account various reasons, during the intubation treatment of PICC cancer patients, the nursing staff will adopt more humane patient care methods to eliminate the psychological burden of the patients, so that the patients are full of confidence in the treatment work and actively cooperate with the medical staff. Adjust the patient's understanding of the disease so that the patient actively fights the disease.

### 4.2. SPSS Statistical Analysis

#### 4.2.1. SPSS Statistical Model Data Analysis

The SPSS statistical model can simultaneously measure the error rate of experimental data and the actual situation. In the process of data analysis, we found that these three prediction models have different degrees of deviation in the hospital's data prediction. Compared with the other two models, the RIMA product model has lower deviations. At this stage of the hospital's statistical forecasting process, SPSS software model forecasting is a popular method. Among them, the ARIMA model combines large-scale analysis methods into random time series analysis, which can make short-term forecasts with high precision. The process of establishing the RIMA model is relatively cumbersome and the calculation process is more complicated, but the prediction results are very good, especially when we predict the number of hospitals, the absolute value of the relative error is relatively small. The comparison table of the predicted values of the three SPSS prediction models on the experimental objects is shown in Table 1, and the comparison chart is shown in Figure 3.

Through the data analysis of the predicted values of the three SPSS prediction models on the experimental objects, a comparison table of the error rates of the predicted values of the three SPSS prediction models on the experimental objects can be obtained, as shown in Table 2.

Figure 4 shows the comparison of the error rate of the three SPSS prediction models on the outpatient volume.

#### 4.2.2. SPSS Statistical Data Inspection and Analysis

Observe the complications of the two groups of patients and their satisfaction with nursing practice. SPSS statistical software is used for the statistical analysis of research data. All data will be analyzed and compared with the test. The general clinical characteristics, tumor characteristics, total effective rate, and toxic reaction differences between the two groups of patients will be compared through *χ*^2^. The *t*-test compares the differences between the means of continuous variables such as age. Several variants were performed using a simulated risk model (Cox regression model), and then the test method was entered.

The occurrence of complications in the observation group who took PICC care is shown in Table 3 and Figure 5.

The occurrence of complications in the control group who took routine infusion care is shown in Table 4 and Figure 6.

In addition to comparing the occurrence of complications between the two groups of patients, it is also necessary to compare and observe the care satisfaction of the two groups of patients. The nursing satisfaction of the observation group and the control group is shown in Table 5 and Table 6.

Through calculation, it can be known that the nursing satisfaction of the observation group was 92.2%, and the nursing satisfaction of the control group was 56.7%. It can be seen that the nursing satisfaction of the observation group was significantly higher than that of the control group.

## 5. Conclusions

PICC is used more and more frequently in nursing solutions, which shows its importance to patients with esophageal cancer. With the advancement of economy and technology, medical technology has improved, and the demand for PICC catheterization technology has also increased. In addition to being higher and more accurate for effective catheterization, efforts must also be increased to avoid complications while minimizing the harm to the patient during treatment. It is necessary to increase effective nursing interventions during PICC nursing. It can improve the treatment effect of patients with esophageal cancer. In this study, PICC is used to care for patients with esophageal cancer, which can effectively improve the patient's physical condition, avoid complications, and have long-term care satisfaction worthy of promotion.

## Figures and Tables

**Figure 1:** PICC catheter diagram in the body (this picture is borrowed from Baidu Encyclopedia).

**Figure 2:** Correlation coefficient *r* and its degree of correlation.

**Figure 3:** Comparison of the predicted values of the three SPSS prediction models on experimental subjects.

**Figure 4:** Comparison of the error rate of the three SPSS prediction models for outpatient volume.

**Figure 5:** The occurrence of complications in the observation group.

**Figure 6:** The occurrence of complications in the control group.

**Table 1:** Comparison table of the predicted values of the three SPSS prediction models on experimental subjects.

Period	Real quantity	Logarithmic model	Exponential smoothing model	RIMA product model
II	27	21	23	25
III	32	27	28	31
IV	31	35	28	33

**Table 2:** Comparison table of error rate of three SPSS prediction models for outpatient volume (%).

Period	Logarithmic model	Exponential smoothing model	RIMA product model
II	22.22	14.81	7.41
III	15.63	12.50	3.13
IV	12.90	9.68	6.45

**Table 3:** The occurrence of complications in the observation group.

Period	Bleeding	Infection	Phlebitis	Total
II	4	1	0	5
III	3	1	1	5
IV	5	2	0	7

**Table 4:** Occurrence of complications in the control group.

Period	Bleeding	Infection	Phlebitis	Total
II	11	4	3	20
III	9	5	2	16
IV	12	5	2	19

**Table 5:** Satisfaction with nursing care of patients in the observation group.

Period	Very satisfied	Satisfaction	General	Dissatisfied
II	7	20	2	1
III	6	23	1	0
IV	6	21	2	1

**Table 6:** Satisfaction with care of patients in the control group.

Period	Very satisfied	Satisfaction	General	Dissatisfied
II	2	15	10	3
III	0	16	9	5
IV	1	17	9	3

## Data Availability

No data were used to support this study.
